# Urgent Transcatheter Arterial Embolization for Wunderlich Syndrome With Hypovolemic Shock Secondary to Ruptured Renal Angiomyolipoma

**DOI:** 10.3389/fsurg.2021.704478

**Published:** 2021-08-13

**Authors:** Maofeng Gong, Zhengli Liu, Haobo Su, Boxiang Zhao, Jie Kong, Xu He

**Affiliations:** Department of Vascular and Interventional Radiology, Nanjing First Hospital, Nanjing Medical University, Nanjing, China

**Keywords:** wunderlich syndrome, renal angiomyolipoma, arterial embolization, embolic materials, interventional radiology

## Abstract

**Purpose:** Wunderlich syndrome (WS) with hypovolemic shock secondary to ruptured renal angiomyolipoma (rAML) represents an urgent condition. Hence, we reported our experience with transcatheter arterial embolization (TAE) using different embolic materials under this condition.

**Methods:** This retrospective study consisted of 22 patients. Embolic materials including particles, microcoils, and liquid embolic agents were selectively used based on the decisions of interventional radiologists. Technical success was defined as the complete occlusion of bleeding vessels on the final renal angiogram. Clinical success was defined as the absence of re-hemorrhage needed for repeat endovascular or surgery treatment after TAE.

**Results:** The articulated materials were used when WS presented without aneurysms; a combination of particulate materials and microcoils or Glubran 2 alone were used for WS with aneurysms. The technical success based on 24 episodes of TAEs in 22 patients was 100% (24 of 24). Repeat TAE was achieved in two patients with hemorrhages re-occurring two days after the initial embolization with microcoils alone. The clinical success was 90.9% (20 of 22). No nontarget embolization or embolization-related complications occurred during the TAE procedure. Of the patients, 27.3% (6 of 22) experienced minor complications of post-embolization syndrome (PES). During a median follow-up time of 34 months, no recurrent hemorrhage that required repeat endovascular or surgical treatment for hemostasis occurred.

**Conclusion:** Urgent TAE with the selective use of different embolic materials is an effective alternative to control WS with hypovolemic shock secondary to ruptured rAML. The condition of presenting with or without aneurysms may determine the embolic materials employed.

## Introduction

Renal angiomyolipoma (rAML) is an uncommon hamartomatous neoplasm of the renal cortex. It consists of tri-phasic tissue with fat, smooth muscle, and abnormal blood vessels in varying proportions, and it usually occurs randomly or in adjunctive with tuberous sclerosis (TSC) (1, 2). Despite being benign, it can possibly grow larger over time, potentially leading to various complications. Hemorrhage is a major complication of rAML that can be severe or life threatening. It is found in more than half of the patients (with tumors size >4 cm) (2, 3). Ruptured rAML may be the most common cause (accounting for 35–40%) of benign neoplasm for Wunderlich syndrome (WS), which is a rare clinical condition classically characterized by the Lenk's triad (flank pain, flank mass, and hypovolemic shock) (4, 5).

Patients presented with ruptured rAML are generally in urgent conditions that require immediate treatment (2, 5). Historically, surgery was the first-line option. However, complete or partial nephrectomy is now thought to be associated with the risk of declining renal function and the loss of renal parenchyma (6). In addition, nephron-sparing surgery is also difficult to perform given the urgent condition and severe tissue adhesion of hemorrhage (7). Therefore, selective nephron-sparing transcatheter arterial embolization (TAE) is currently the treatment of choice for rAML. It may avoid emergent radical surgery (2, 5–7) and have prophylactic effects in preventing future hemorrhage (8).

TAE for WS with hypovolemic shock secondary to ruptured AML is perceived as a more formidable task because of the usual urgency of the condition (7). Embolic materials used mainly involved particles [such as gelatin sponge particles (GSP), polyvinyl alcohols (PVA), microparticles, and microsphere], coils, and liquid agents (such as ethanol, ethiodized oil, ethylene vinyl alcohol copolymer, etc.) (2, 6–9). Each material has its specific benefits and drawbacks, and there are no prospective and comparative studies that establish strong recommendations on which one to choose (9). In this paper, we present our experience with TAE using different embolic materials, alone or in combination, to treat WS with hypovolemic shock secondary to ruptured rAML.

## Methods

### Study Design

This retrospective study was approved by both our institutional review board and by the written consent of patients. This study reviewed patients with WS secondary to rAML between March 2012 and March 2020 at a single academic university hospital, including 22 consecutive patients with hypovolemic shock who subsequently experienced 24 episodes of TAEs. Of these, two patients received additional embolization with microspheres in the second procedure. CT scans confirmed that these patients had WS, and that their kidneys had lost the normal morphological structure: the density of internal rAML structures was heterogeneous, including multiple low-density (fatty tissue) areas. A contrast-enhanced CT scan was used to identify the entity of the hemorrhage and eliminate other underlying causes of WS. The diagnosis of WS with hypovolemic shock secondary to ruptured AML was based on clinical manifestations, decreased hemoglobin levels, and specific radiologic characteristics on CT scan findings. Data collected from the medical records included the control of hypovolemic shock (technical success and clinical success), the varieties and volumes of embolic material, complications, preintervention and postintervention renal function, and AML size.

### Transcatheter Arterial Embolization Procedure

The embolic materials employed in the present study were GSP (Alicon Pharm, Ltd., Hangzhou, China), PVA (Cook, Bloomington, IN, USA), microspheres (Embosphere; Merit, Rockland, MA, USA), microcoils (Cook, Bloomington, IN, USA), or Glubran 2^®^ (N-butyl-2 cyanoacrylate; GEM, Viareggio, Italy). The benefits and potential risks of TAE were explained to the patients and/or their relatives, and detailed informed consent was obtained from all patients.

The choice of embolic materials was proposed by interventional radiologists in our center. Two interventional radiologists with 20-year experience performed all procedures. To identify and localize active bleeding sites and feeder arteries of rAML, before embolization, an accurate overview angiogram was performed under local anesthesia with a 5-French (F) selective Simon catheter (Radifocus Angio-graphic Catheter; Terumo, Leuven, Belgium) through a 5-F introducer (Radifocus Introducer II Introducer Sheath; Terumo, Leuven, Belgium) into the right femoral artery. After identifying the arterial tumor feeders and bleeding site, a compatible 2.4-F microcatheter (Progreat; Terumo, Leuven, Belgium) was then coaxially positioned, ensuring that the microcatheter tip was as close as possible to the target bleeding site. Under fluoroscopy control, GSP, PVA, microspheres, or Glubran 2^®^ was injected as slowly as possible using thumb pressure and adjusted according to embolic material propagation in the bleeding artery and target arterial flow speed. If possible, it was continued until the feeding bleeding vessels were completely occluded to avoid undesired embolization of normal arterial branches and reduce infarcted renal parenchyma loss as much as possible. For patients without aneurysms, GSP, PVA, or microspheres were used solely. For patients with aneurysms, GSP or PVA was used, followed by microcoils according to the diameter of target vessel, to embolize the feeder artery trunk. For patients who underwent failed TAE with microcoils alone for pseudoaneurysms, rescue TAE with microspheres was performed. Glubran 2 was successfully employed as a sole embolic material in patients under severe coagulopathic condition [defined by an abnormal value for prothrombin time, activated partial thromboplastin time, and/or a reduced platelet count (<50 × 10^9^/L)]. At the end of embolization, the microcatheter was withdrawn, and a final renal angiogram through the 5-F Simon catheter was performed to evaluate vessel occlusion. Patients with post-embolization syndrome (PES), including aggravation of flank pain and low-grade fever (37.6–37.9°C), were given supportive treatment (tramadol injection for analgesia and ice bag for physical cooling temperature) until the symptoms disappeared.

### Definitions of Efficacy, Safety, and Follow-Up

The efficacy of TAE included both technical and clinical evaluations. Technical efficacy was defined as the complete occlusion of target bleeding vessels on the final renal angiogram, while the clinical efficacy was defined as the absence of re-hemorrhage needed for repeat endovascular or surgery treatment after TAE (10). The safety of TAE was evaluated based on complications that occurred mid-TAE, especially clinically or technically adverse events mid-intervention. The renal function was assessed by comparing serum creatinine (Scr) and blood urea nitrogen (BUN) levels after one week of preintervention. One week after treatment, renal function was retested and compared with the function before TAE. During the follow-up, CT and/or Doppler Ultrasound on the abdomen and clinical evaluations were performed on an outpatient basis for all patients on the first, third, and sixth months and at 6-month intervals thereafter or sooner when clinically indicated. Any instances of recurrent bleeding or post-TAE complications were recorded.

### Statistical Analyses

*SPSS* statistical software package (version 23.0; *SPSS* statistical software, Chicago, Illinois, USA) was used for all statistical analyses. Continuous variables were expressed as the means ± standard deviation. Qualitative variables were presented as percentages. When assessing the correlation between pre-intervention and post-intervention variables, a paired *t-*test was used. Findings with a *P* value < 0.05 were deemed statistically significant.

## Results

The demographic, clinical characteristics, embolic materials used, and outcome of the patients are shown in Table 1. The study included 12 female and 10 male patients aged 37–90 years (mean, 56.3 ± 16.3 years). Two patients (9.1%) were diagnosed with a TSC in other hospitals. All patients presented with hypovolemic sock, accompanied with flank pain (81.8%) and hematuria (59.1%).

**Table 1:** Patients underwent TAE with different materials for Wunderlich syndrome (WS) with hypovolemic shock secondary to ruptured renal AML.

**Patient No**.	**Gender/Age**	**Symptoms (except** **hypovolemic sock^a^)**	**Whether** **with Aneurysm**	**Embolization** **Site**	**Sessions/** **(Embolic materials)**	**GSP/PVA**		**Microcoils**		**Success^b^**
						**Size (μm)**	**Numbers**		**Size (mm)**	**Numbers**
1	M/41	Flank pain	No	RUP	I/GSP	560–710	50 mg	-	-	Yes
2	M/48	Hematuria	No	LUP	I/GSP	560–710	100 mg	-	-	Yes
3	F/61	Flank pain, Hematuria	No	RMP	I/Microspheres	500–700	1 ml	-	-	Yes
4	M/40	Flank pain	Yes	LUP	I/Glubran 2	1:7	1.4 ml	-	-	Yes
5	F/37	Flank pain, Hematuria	Yes	LLP	I/(PVA+Microcoils)	350–560	40 mg	2*20, 2*30, 3*30	3	Yes
6	F/64	Flank pain	Yes	RLP	I/(PVA+Microcoils)	350–560	40 mg	2*20	3	Yes
7	M/42	Flank pain, Hematuria	Yes	LMP	I/(GSP+Microcoils)	700–900	30 mg	3*30, 4*30, 5*50	3	Yes
8	F/73	Flank pain	Yes	LUP	I/(PVA+Microcoils)	350–560	50 mg	2*30, 3*30, 4*20, 4*30	4	Yes
9	F/90	Hematuria	No	RMP	I/PVA	560–710	70 mg	-	-	Yes
10	F/74	Flank pain, Hematuria	Yes	LLP	I/Microcoils; II/Microspheres	100–300	1 ml	2*20, 3*20	2	I No; II Yes^c^
11	M/51	Flank pain	Yes	RLP	I/Glubran 2	1:3	0.9 ml	-	-	Yes
12	M/43	Flank pain	No	RUP	I/GSP	560–710	40 mg	-	-	Yes
13	M/59	Flank pain, Hematuria	No	LLP	I/Microspheres	500–700	1 ml	-	-	Yes
14	M/39	Flank pain	Yes	LUP	I/Glubran 2	1:7	1.2 ml	-	-	Yes
15	F/44	Hematuria	No	RMP	I/GSP	560–710	100 mg	-	-	Yes
16	F/41	Flank pain, Hematuria	Yes	LUP	I/(PVA+Microcoils)	350–560	40 mg	2*20, 3*30, 3*30	3	Yes
17	F/72	Flank pain, Hematuria	Yes	LUP	I/Microcoils; II/Microspheres	100–300	1.1 ml	2*30, 3*20	3	I No; II Yes^c^
18	M/43	Flank pain, Hematuria	Yes	LUP	I/(GSP+Microcoils)	700–900	20 mg	3*20, 4*30, 5*50	3	Yes
19	F/89	Flank pain	No	LUP	I/PVA	560–710	50 mg	-	-	Yes
20	F/72	Flank pain, Hematuria	Yes	RMP	I/(PVA+Microcoils)	350–560	60 mg	2*20, 3*20, 4*20, 4*30	4	Yes
21	F/60	Flank pain	Yes	RLP	I/(PVA+Microcoils)	350–560	30 mg	2*30	3	Yes
22	M/56	Hematuria	Yes	RLP	I/Glubran 2	1:3	0.8 ml	-	-	Yes

*TAE, transcatheter arterial embolization; WS, Wunderlich syndrome; AML, angiomyolipoma; F, female; M, male; LUP, left upper pole; LLP, left lower pole; RUP, right upper pole; RMP, right middle pole; RLP, right lower pole; GSP, gelatin sponge particles; PVA, polyvinyl alcohol*.

a *All patients encountered hypovolemic shock symptom*.

b *Success included technical and clinical success*.

c *Secondary TAE was achieved in these patients owning to hemorrhage recurrence 2 days after initial TAE. Technical success was achieved. The second clinical success was achieved*.

Twenty-two patients received a total of 24 episodes of TAEs. Of these, 8 patients (36.3%) without aneurysms in neoplasm underwent TAE using GSP (560–710 μm), microspheres (500–700 μm), and PVA (350–560 μm) alone. Eight patients (36.3%) with proven aneurysm formation in neoplasm underwent median 40 mg initial PVA (350–560 μm) or GSP (700–900 μm) embolization of bleeding sites, and additional total 31 microcoils (range, 2–5 mm × 20–50 mm) in the feeder artery trunk in a single session. Two patients (9.1%) identified with pseudoaneurysms in AML underwent microcoils (2 mm × 20 mm and 3 mm × 20 mm; 2 mm × 30 mm and 3 mm × 20 mm) embolization in feeder trunk vessel alone; hematuria suddenly occurred two days following TAE, accompanied with tachycardia and decreased blood pressure, and disappeared after receiving rescue TAE with microspheres (100–300 μm, Figure 1). Glubran 2 was successful employed as a sole embolic material in 4 patients (18.2%) under severe coagulopathic condition (Figure 2), the concentration ratios were 1:3 and 1:7, and total volume injected was median 1.1 ml. Final angiography revealed complete occlusion of all targeted vessels, and the technical success of embolization was achieved in 100% of patients (22 of 22).

**Figure 1:** Collateral feeding arteries formed lead to clinical failure after embolization using microcoils alone. **(a)** Right renal arteriography reveals emerging collateral feeding arteries (white arrow) arising from adjacent artery supply the distal portion of the initial bleeding artery; **(b)** The hemorrhage disappears following repeat embolization with microspheres (100–300 μm).

**Figure 2:** A patient who encountered Wunderlich syndrome (WS) secondary to ruptured renal angiomyolipoma (rAML) underwent transcatheter arterial embolization (TAE) using Glubran 2. **(a)** The left renal overview arteriography revealed a dysplastic and aneurysmal artery (white arrow); **(b)** Thumb pressure angiogram through the microcatheter demonstrated rupture of the renal parenchyma and spilling of the contrast agent (white arrow); **(c)** The mixture of Glubran 2 and ethiodized oil (concentration ratio 1:7) was injected as slowly as possible into the bleeding target arterial, cast filling dysplastic, and aneurysmal arteries (white arrow); **(d)** Completion arteriography after TAE with Glubran 2 demonstrating AML devascularization and maximum preservation of the normal renal parenchyma.

All patients in pre-intervention encountered hypovolemic shock with mean systolic pressure 80.8 ± 9 mmHg. All patients also experienced stable hemodynamic status and an increase in blood pressure following TAE to 115.9 ± 11.3 mmHg (*t* = −13.1, 95% CI −41.1 to −29. 1, *P* < 0.001). Their anemia symptoms improved after blood transfusion and TAE treatment. The clinical success was achieved in 90.9% of patients (20 of 22). Twenty patients were freed from re-hemorrhage after receiving TAE, and repeat TAE with microspheres was achieved in two patients due to hemorrhage re-occurring two days after initial embolization with microcoils alone.

No non-target embolization or embolization-related complications occurred during the TAE. Six patients (27.3%) experienced minor complications of PES, including aggravation of flank pain and low-grade fever (37.6–37.9°C). They received conservative treatment for 3 days and recovered without permanent complications. The amount of contrast material and duration of fluoroscopy were 49.8 ± 11.8 ml (320 mg I/ml; range, 30–70 ml) and 22.0 ± 5.0 min (range, 15–30 min), respectively. There were no significant changes in Scr and BUN levels pre-intervention and one week after embolization (Figure 3) (*P* > 0.05). The renal function information was assessed *via* the evaluated glomerular filtration rate (eGFR), and mean levels before and one week after TAE were 83.2 ± 29.9 ml/min and 80.7 ± 31.5 ml/min, respectively, which was not a significant difference (*t* = 0.5, 95% CI −6.6 to 11.5, *P* > 0.05).

**Figure 3:** The progression of renal function during a six-month follow-up period. No significant changes in serum creatinine and urea nitrogen level preintervention and postintervention during follow-up period (*P* > 0.05).

With a median of 34 months follow-up, neither hypovolemic shock due to hemorrhage nor recurrent further ruptures of the tumor were observed. Surgical treatment was avoided in all patients, and renal function remained stable during the follow-up period, with no significant change in Scr and BUN levels noted in individual patients. The tumor size of the rAML was observed using CT alone and CT adjunctive with ultrasound (US) in 8 patients, showing that the mean maximum diameter of the renal tumor on CT scan in the 22 patients reduced from 60.5 ± 12.7 mm to 45.8 ± 13.6 mm at the last follow-up visit, which was significantly smaller (*t* = 7.77, 95% *CI* 10.4 to 18.8, *P* < 0.001, Figure 4). The median duration of perirenal hemorrhage due to WS was average 3 months (Figure 5).

**Figure 4:** The CT images of renal angiomyolipoma (rAML) size in preintervention and postintervention after transcatheter arterial embolization (TAE) (the same patient as in Figure 2) were showed. An inhomogeneous endophytic renal mass with low-attenuating areas of intra-tumoral fat. **(a–f)** CT images obtained at pre-TAE, and at follow-up period of 1 week, 1 month, 3 months, 6 months, and 12 months. A significant reduction in rAML size was depicted.

**Figure 5:** The CT findings of renal hemorrhage size owing to Wunderlich syndrome (WS) pre- and post-transcatheter arterial embolization (TAE) (the same patient as in Figure 2) were listed. High-attenuating hemorrhagic areas were seen around the kidney. **(a–f)** CT image obtained at pre-TAE, and at follow-up period of 1 week, 1 month, 3 months, 6 months, and 12 months. A significant reduction in hemorrhage size was observed.

## Discussion

WS, also known as spontaneous renal hemorrhage, was first described by Wunderlich in 1,856 with a condition of spontaneous renal hemorrhage with dissection of blood into the subcapsular and/or perinephric spaces (3, 4). Literature showed that 83% of cases presented with acute onset of flank pain, 19% had hematuria, and 11% had symptoms and signs of hypovolemic shock (11). The presence of all three symptoms is uncommon (12). Enlarged rAML is at a high risk of rupture due to abnormal elastin-poor tortuous vessels predisposed to aneurysm formation causing WS, and heterogeneous proportion is often altered on CT by hemorrhage within the lesion and perirenal hemorrhage (2, 3, 11). Conservative treatment for WS may be considered in hemodynamically stable patients; however, WS within the context of hypovolemic shock may require an urgent management strategy, for which there is no clear consensus in the literature regarding the embolization technique and the choice of embolic materials. Thus, we implemented the method of TAE with different embolic materials under this condition.

In a recent systematic review of WS, only 102 cases were presented in 79 pieces of literature, which is insufficient for studying the WS treatment (11). Although our study population of 22 patients is not particularly big, we have shown that urgent TAE has been effective for WS with hypovolemic shock secondary to ruptured rAML. Patients who suffered from WS with hemodynamic instability avoided further surgery after urgent TAE, and the perirenal hemorrhage of WS could be absorbed within three months during follow-up, without nephrectomy or nephron-sparing surgery. The use of sole microcoils in TAE for rAML has been debatable, as collaterals can potentially form occlusion and make further embolization difficult when hemorrhage re-occurrs (13, 14). In our study, two patients required repeat embolization with microcoils as the only embolic materials. Fortunately, rescue treatment was sucessful achieved with small microspheres (100–300 μm). Although pulmonary or renal dysfunction were reported in literatures (2, 15), whereas, was not observed in the present study. WS with hypovolemic shock secondary to AML are benign tumors with a ruptured vascular component; thus, they behave like, and must be treated as, part-bleeding site and part-aneurysm (8). Therefore, we used particles to achieve hemorrhage stasis. Since the aneurysm remains pressurized and at risk of rupture, coil placement was the most efficient technique (13, 14); combination of occlusion of the distal vascular bed with particles followed by microcoils occlusion of the arterial inflow to prevent retrograde filling of the aneurysm have been used in the present study.

Glubran 2, a modified N-butyl-2 cyanoacrylate, seems to be a potent alternative liquid embolic agent used for rAML to stop hemorrhage. In our study, four patients with hypovolemic shock WS secondary to rAML under coagulopathic condition underwent successful hemostasis. Before TAE, in order to improve presentation, Glubran 2 was thoroughly mixed with ethiodized oil. Concentration ratios were 1:3 and 1:7, depending on the arterial flow speed and the distance between the microcatheter tip and the bleeding site. This material appears to be a promising alternative under the condition of coagulopathy, even though complete hemostasis is difficult to achieve. Polymerization can occur immediately upon contact with blood, leading to instant and complete vessel occlusion. Thus, Glubran 2 has advantages in coagulopathy due to its abilities of penetration and the formation of an intravascular cast extending from the smaller, distal tumor vasculature to the proximal, larger blood supply, along with its predictability and controllability (16).

In our study, the maximum diameter of AML before TAE was 60.5 ± 12.7 mm. With 34 months of follow-up, the maximum diameter of the tumor decreased to 45.8 ± 13.6 mm, which was significantly smaller. Vessels on the tumor appeared to have reduced in size disproportionally compared to the fat component, which explains the variability in overall reduction of the AML sizes. The fat component appeared to be relatively insensitive to embolization, whereas the vessel components responded well, which indicated that the tumor shrinkage was mainly due to the large reduction in vessel components and smooth muscle atrophy (17). Because of the different proportions of blood vessels, smooth muscles, and fat content in different tumors, AML in our study were completely occluded. Therefore, the size reduction correlated with the success of the procedure and showed significantly reduced volume.

In terms of the safety of TAE with different embolic materials for WS secondary to rAML, no complications occurred during the mid-procedure related to TAE. PES, which is characterized as the most frequent complication of embolization by fever and flank pain, occurs in up to 36% of cases (18). In the present study, 27.3% of patients experienced PES that presented as aggravation of flank pain and low-grade fever, which were treated conservatively; all the patients recovered without permanent complications. It was demonstrated that AML would shrink with liquefactive necrosis and tend to induce abscess formation post-TAE (11). Additionally, there were no local infection cases in our study with these modalities of embolization. The preservation of renal function was a crucial factor in renal embolization in this population given the benign nature of the disease, the average age of diagnosis, and the emerging body of evidence that has been associated with an improved overall survival (7). In our study, renal function was not affected. Therefore, we consider that TAE does not increase risk of complications.

Previous studies on the treatment of WS are mostly anecdotal case reports. To the best of our knowledge, our study may be the sole study regarding embolization using different embolic materials for the treatment of WS due to ruptured rAML. This may offer experience for future researchers. However, our study had several limitations. First, it was performed at a single center with a small patient pool. Second, no comparative analysis in different embolic materials was made, which could be an interesting issue. Third, cases in our study were confirmed without the pathology before TAE due to an emergent hypovolemic shock condition; whereas rAML was clearly diagnosed by three senior radiologists based on typical CT scan.

In conclusion, urgent TAE with the selective use of different embolic materials play an important role in controlling the WS with hypovolemic shock secondary to ruptured rAML. It causes little damage to renal function, results in moderate complications, and reduces the need for immediate radical surgery. We preferred particulate materials for WS without aneurysms, a combination of particulate materials and microcoils, or Glubran 2 alone for WS with aneurysms. Studies over a larger population are required to determine these conclusions of WS with hypovolemic shock secondary to ruptured rAML.

## Data Availability Statement

The original contributions presented in the study are included in the article/supplementary material, further inquiries can be directed to the corresponding author/s.

## Ethics Statement

The studies involving human participants were reviewed and approved by the institutional review board (IRB) of the Nanjing First Hospital, Nanjing Medical University (Nanjing, China). The patients/participants provided their written informed consent to participate in this study.

## Author Contributions

MG contributed to project development, data collection, manuscript writing/editing. ZL, HS, and BZ contributed to project development, data collection, data analysis. BZ manuscript editing. JK and XH contributed to project development. All authors contributed to the article and approved the submitted version.

## Conflict of Interest

The authors declare that the research was conducted in the absence of any commercial or financial relationships that could be construed as a potential conflict of interest.

## Publisher's Note

All claims expressed in this article are solely those of the authors and do not necessarily represent those of their affiliated organizations, or those of the publisher, the editors and the reviewers. Any product that may be evaluated in this article, or claim that may be made by its manufacturer, is not guaranteed or endorsed by the publisher.
